The article "Security Analysis of Social Network Topic Mining Using Big Data and Optimized Deep Convolutional Neural Network" was published in 2022. Journal: Comput Intell Neurosci.

# Security Analysis of Social Network Topic Mining Using Big Data and Optimized Deep Convolutional Neural Network

**DOI:** 10.1155/2022/8045968

**Published:** 2022-09-23

**Authors:** Kunzhi Tang, Chengang Zeng, Yuxi Fu, Gang Zhu

**Affiliations:** ^1^College of Engineering & Computer Science, The Australian National University, Canberra 2615, Australia; ^2^School of International Education, Zhejiang Normal University, Jinhua 321004, China; ^3^Department of Science and Technology, Beijing Normal University-Hong Kong Baptist University United International College, Zhuhai 519087, China; ^4^Chinese Academy of International Trade and Economic Cooperation, Beijing 100000, China

## Abstract

This research aims to conduct topic mining and data analysis of social network security using social network big data. At present, the main problem is that users' behavior on social networks may reveal their private data. The main contribution lies in the establishment of a network security topic detection model combining Convolutional Neural Network (CNN) and social network big data technology. Deep Convolution Neural Network (DCNN) is utilized to complete the analysis and search of social network security issues. The Long Short-Term Memory (LSTM) algorithm is used for the extraction of Weibo topic information in the memory wisdom. Experimental results show that the recognition accuracy of the constructed model can reach 96.17% after 120 iterations, which is at least 5.4% higher than other models. Additionally, the accuracy, recall, and *F*1 value of the intrusion detection model are 88.57%, 75.22%, and 72.05%, respectively. Compared with other algorithms, the model's accuracy, recall, and *F*1 value are at least 3.1% higher than other models. In addition, the training time and testing time of the improved DCNN network security detection model are stabilized at 65.86 s and 27.90 s, respectively. The prediction time of the improved DCNN network security detection model is significantly shortened compared with that of the models proposed by other scholars. The experimental conclusion is that the improved DCNN has the characteristics of lower delay under deep learning. The model shows good performance for network data security transmission.

## 1. Introduction

In recent years, the Internet technology has made unprecedented progress with the continuous acceleration of the globalization process [1]. The number of smart grid terminals has increased, big data, cloud computing, and other technologies have been applied in various fields, and the amount of data on the Internet has been exploded [2]. The Internet has gradually entered the era of big data with the new features of high value and high transmission speed. Data provides more support for people to find and extract useful information. The cross-age progress of the Internet has made social networks larger and more diverse in forms. Various social networks, such as QQ, WeChat, and Weibo, have completely changed the life [3].

The article "Security Analysis of Social Network Topic Mining Using Big Data and Optimized Deep Convolutional Neural Network" was published in 2022. Journal: Comput Intell Neurosci.

However, the development of science and technology is a two-edged weapon. The rapid technological progress brings not only a new way of life but also the subsequent network information security issues [4]. In social networks, users are often threatened by network security issues including network attacks, private data leakage, misuse, and theft of confidential information. In the current network information security monitoring system, there are many methods and strategies for managing network information security [5]. However, all these methods have varying degrees of deficiencies in terms of security and operability when facing a huge amount of data. They cannot detect security topic information on the network in time, especially the effective information contained in the massive data of social networks. Traditional information search technology is difficult to search and extract in time [6]. Therefore, to ensure data and information security, timely and effective social network security topic mining and analysis models are particularly important for the development of information security and network security [7].

To sum up, in today's diverse social networks, it is particularly important to mine and analyze the security topic data on social networks and meanwhile ensure the security of users' social network information and avoid the leakage and data loss of users' private data [8]. At present, the main problem is that the topics discussed on social networks are mixed, and the inadvertent behavior of users on social networks may leak their private data and threaten their privacy. The main contribution of the research lies in the establishment of a network security topic detection model by combining deep convolutional neural network (DCNN) and social network big data technology. The main innovation lies in the use of DCNN to complete the analysis and search of social network security issues. The Long Short-Term Memory (LSTM) is used to extract Weibo topic information in the memory wisdom algorithm. This is the uniqueness and novelty of research and provides an experimental reference for the subsequent improvement of the topic security and data transmission performance of social networks.

## 2. Recent Related Work

### 2.1. Research Status of DCNNs

In recent years, the classification accuracy of Deep Neural Network (DNN) and convolutional neural network (CNN) has begun to significantly improve with the increasing network structure and the comprehensive improvement of hardware performance [9], as the neural network model of the multilayer network structure. The neural network model has been widely used in many fields, such as system intrusion detection and images remote sensing recognition [10]. Rm et al. used DNN to study benchmark intrusion detection in the medical IoT environment, and the results showed that the performance of the DNN model was more accurate than the original machine learning algorithm, and the time complexity was reduced by 32% [11]. Devan and Khare used the softmax classifier to classify network intrusions under the Tensor flow framework through DNNs, and the results showed that the model was better than the shallow machine learning algorithm of the original data set [12]. Chen et al. used an improved CNN architecture to evaluate and calibrate the pollution degree of agricultural irrigation water resources and improve the accuracy of near-infrared prediction [13]. Igarashi et al. used DCNN (AlexNet) to predict and study the degree of cancer invasion on endoscopic images of the upper gastrointestinal tract. The accuracy rates of the trained and validated data sets are, respectively, 99.3% and 96.5% [14]. Kattenborn et al. used deep learning CNNs to extract vegetation attributes from remote sensing images. Those improve the spatial resolution of vegetation remote sensing data [15]. Awais et al. studied the classification of mixed and awake states of newborns based on DCNN and support vector machine algorithms. Its accuracy rate reaches 93.8% [16]. In summary, CNN and DCNN have been widely used in computer vision in various fields.

The article "Security Analysis of Social Network Topic Mining Using Big Data and Optimized Deep Convolutional Neural Network" was published in 2022. Journal: Comput Intell Neurosci.

### 2.2. Status of Social Network Security Issues

With the rapid development of social networks, the personal privacy leakage of users has become more and more serious. The private information of users in social networks is illegally collected and used. Many scholars have conducted related researches to solve the security protection problems of social networks. Alshaikh et al. proposed a privacy measurement algorithm on the degree of adjacency to achieve the level of data availability and privacy protection “trade-off” based on the differential privacy model, combined with clustering and randomization algorithms [17]. Zhan and Tao studied the security protection technology and security protection mechanism under the 5th Generation Mobile Communication Technology (5G) network [18]. Maragatham et al. found that the trust-based photo-sharing component can help solve the security problems in the photo-sharing process of social platforms through simulation experiments [19]. Meanwhile, the anonymization of pictures should be represented with the edge characterized by the distributor.

The article "Security Analysis of Social Network Topic Mining Using Big Data and Optimized Deep Convolutional Neural Network" was published in 2022. Journal: Comput Intell Neurosci.

The security issues of social networks are still at a basic stage by analyzing the research of the abovementioned scholars. Few scholars apply DCNNs to the topic mining and analysis of social network security. Therefore, the use of DCNN to construct social network information security and intrusion detection models has extremely important practical guiding significance for the analysis and prediction of network information security under the trend of increasing information security risks of social networks [20].

## 3. Weibo Security Topic Mining and Security Analysis on DCNN

### 3.1. Topic Mining and Demand Analysis of Social Network Security

Weibo is one of the social networking platforms that people use the most in their daily lives. The information on Weibo can not only describe people's daily life, but also the opinions and experiences of different groups of people on a certain item. The topic of Weibo has become an important basis for reflecting popular social topics [21]. This research can identify and monitor important topics that affect network security from Weibo. The most important thing is to collect all Weibo information on the topic in time after the incident. To collect topic information comprehensively, it is necessary to transform the messages sent by users into a topic model. After the feature expression of Weibo is obtained in the experiment, the DCNN model is used to train and learn the deep semantic information in Weibo, and the system will accurately identify and detect the topic feature expression of Weibo [22].  Figure 1 shows the mining of topic data on social networks. The social network data extracted from the user's mobile phone client and computer terminal are filtered by the Internet, stored in a big data center, and extracted and analyzed through the data center when needed.

### 3.2. Weibo Search Ranking and Topic Feature Mining and Extraction

Weibo search ranking is playing an increasingly important role in Weibo exploration and analysis [23]. As a hot research topic, Weibo search is also widely used by academic backgrounds and industries. The main content of the Weibo search is divided into two parts: extraction of Weibo features and research on Weibo topics [24]. The extraction of Weibo features refers to the analysis of the characteristics of Weibo social relations and the temporal and spatial characteristics of Weibo on the micro-meaning of Weibo text information, unifying the content of Weibo blogs, eliminating the semantic gap between media, and performing images and videos and unified extraction of multimedia information. Weibo topic research is to strengthen user search terms by inputting the user's search intent, combining semantic expansion and the expansion of the knowledge base, and implementing a classification model on Weibo features.

The article "Security Analysis of Social Network Topic Mining Using Big Data and Optimized Deep Convolutional Neural Network" was published in 2022. Journal: Comput Intell Neurosci.

In the Weibo search, the most important thing is the related classification, which combines all the features extracted above, and obtains the similarity between the Weibo message to be matched and the user request according to the classification template and returns the search result [25]. The quality of the classification template will affect the user's search experience. The classification template directly determines the order in the search results to study the network, and users tend to pay special attention to the first tweet in the search results. Therefore, the question about the Weibo information at the top of the search results can satisfy the user's needs in terms of information, and the search directly determines the user's search experience. The classification model has played an important role in the Weibo research framework for many years.

Weibo information classification process: extract Weibo features from Weibo information data, select learning methods, learn classification models, and form the weight of each feature [26]. The linear combination used to generate the classification function can be expressed as follows:

(1) $$\begin{array}{c} f\left(x_{i}\right)=\overset{\;|\;F\;|\;}{\underset{j=1}{\sum }}w_{j}*t_{j}\text{,} \end{array}$$

*x*_*i*_ represents the *i*th feature of *t*_j_, *w*_j_ represents the weight value of the *j*th feature in the ranking function, and *F* is the feature set. On the ranking model, the Weibo topic information related to the query sentence will be returned to the search result. The overall feature extraction structure is shown in Figure 2.

### 3.3. Weibo Security Topic Detection on Hidden Dirichlet Distribution

Because Dirichlet distribution has good conjugation and aggregation, it is widely used in the field of deep learning [27]. The Dirichlet distribution is used to mine and analyze the probability distribution of document topics by using common appearance features in the text [28]. Since Dirichlet distribution is an unsupervised learning algorithm, it can easily realize vectorized representation and modeling of text. Here, the trained model is used to extract the topic detection features of the text, the Weibo detection message is used as the topic distribution vector, and the Gibbs sampling algorithm is used to sample the distribution of lexical items. The Gibbs sampling is defined as follows:

(2) $$\begin{array}{c} P\left(z_{i}=k\left|z_{i}\right.,w\right)\theta_{m,k}*\varphi_{k}\text{,} \end{array}$$

(3) $$\begin{array}{c} \varphi_{ki}=\frac{n_{k,i}+\beta_{t}}{\overset{n}{\underset{i=1}{\sum }}\left(n_{k,i}+\beta t\right)}\text{.} \end{array}$$

Equation (2) is the process of document generation, which means that when the *m*th document is generated, the topic number of the *n*th word of the document is first generated from the document distribution matrix. Formula (3) is the process of document word generation, which represents the process of generating the *n*th word of the *m*th document in the thesaurus.

The article "Security Analysis of Social Network Topic Mining Using Big Data and Optimized Deep Convolutional Neural Network" was published in 2022. Journal: Comput Intell Neurosci.

The Dirichlet distribution is the foundation of digital image processing. In the signal analysis and processing link, Fourier Transform is used to transfer the signal from the time domain to the frequency domain. The frequency domain is used to process the signal to more accurately analyze the composition of the signal frequency, laying the foundation for the filtering operation. It is transferred from the spatial domain to the frequency domain after the Fourier transform of the image. Therefore, the image is subjected to Fourier Transform operation. This is very important in the field of digital images. It is the basis of image feature extraction and the basic necessary condition for image edge detection and filtering and noise reduction. The DNN Weibo topic detection algorithm and DCNN's Weibo security topic detection are used to verify the effectiveness of the security topic mining model.

### 3.4. Weibo Topic Detection on DNN

The neural network-based Weibo topic detection method requires the detection object as a classification task [29]. Different from the previous vector machine model supported by the vocabulary unit as the Weibo text vector, the neural network method will extract the latent semantic features of the Weibo text quantization process, and then use the Weibo text vector to form multiple classifiers to supplement the Weibo topic detection Model formation. The research quantifies the text through neural detection of Weibo topics, which has strong linear separability. The framework of the method for detecting Weibo topic objects on neural networks is shown in Figure 3. In the preprocessing part, the text of Weibo is mainly processed for word classification, word banning, and high-frequency word deletion.

### 3.5. Weibo Security Topic Detection Model on DCNN

#### 3.5.1. Long Short-Term Memory (LSTM) Network

A recurrent neural network (RNN) uses short-term information during the training process or makes the model lose the long-term training results. To solve this problem, the research uses the LSTM network structure [30]. In the LSTM network, the threshold structure is introduced into the “forget” and “memory” functions. During training, the threshold structure selectively transmits information to the network so that implicit long-term information can be transmitted during the formation. The vector words formed by the LSTM network can better express the depth of semantic information implicit in the semantic information in the text and obtain more representative vector words of text features, as shown in the following equations.

(4) $$\begin{array}{c} i_{t}=\left(W_{x,i}x_{t}+W_{z,i}Z_{t-1}+b_{i}\right)\text{,} \end{array}$$

(5) $$\begin{array}{c} f_{t}=\left(W_{x,f^{x}t}+W_{z,f^{z}t-1}+b_{f}\right)\text{,} \end{array}$$

(6) $$\begin{array}{c} o_{t}=\left(W_{x,o^{x}t}+W_{z,o^{z}t-1}+b_{o}\right)\text{,} \end{array}$$

(7) $$\begin{array}{c} g_{t}=\tanh\left(W_{x,m^{x}t}+W_{z,m^{z}t-1}+b_{g}\right)\text{,} \end{array}$$

(8) $$\begin{array}{c} m_{t}=f_{t}\circ m_{t-1}+i_{t}\circ g_{t}\text{,} \end{array}$$

(9) $$\begin{array}{c} z_{t}=o_{t}\circ \tanh m_{t}\text{,} \end{array}$$

*m*_*t*_ represents the value *m*_*t*−1_ of the last iteration and the unit function value of the input *x*_*t*_. Pass the vector *o*_*t*_ to all connected layers, and finally, calculate the output value with *z*_*t*_. Meanwhile, *m*_*t*_ indicates the iteration vector representing the number of model training times, which is passed to the next training as part of the input vector for the next iteration. *W* is the weight matrix. *b*_*∗*_ is the bias vector, which is the training parameter of the neural network. *u*∘v represents the dot product operation between the two.

The article "Security Analysis of Social Network Topic Mining Using Big Data and Optimized Deep Convolutional Neural Network" was published in 2022. Journal: Comput Intell Neurosci.

#### 3.5.2. Use the Long and Short Temporal Memory Network to Obtain the Deep Semantic Features of the Weibo Text

On the LSTM sequence memory unit, the construction of the neural network mechanism is shown in Figure 4.

To limit the transmission of the parameters of the neuron network, the maximum number of expansion steps is set as 32, which means that the neuron network will restart after the network is expanded 32 steps forward. A series of Weibo topic data is used as the input of RNN, which predicts the next word and updates the neural network settings according to the prediction accuracy. The LSTM state vector of each iteration step of the neural network is used as the corresponding word vector input to form a neural network until the network converges to the specified maximum number of iterations.

Meanwhile, each Weibo has a start character and an end character. The LSTM state vector corresponding to the formation step of the neural network of the ending character can be expressed as a Weibo vector. After using text corpus data to form a RNN, the proposed method can obtain the Weibo word vector that represents the feature of the Weibo text. This vector representing the text features of Weibo can be used to represent the words in Weibo and apply them to subsequent Weibo search tasks and Weibo topic detection.

The article "Security Analysis of Social Network Topic Mining Using Big Data and Optimized Deep Convolutional Neural Network" was published in 2022. Journal: Comput Intell Neurosci.

#### 3.5.3. Vectorized Representation of Weibo Text

The first step in implementing a Weibo topic object detection model on a DCNN is to quantify Weibo text. The quantification method of Weibo text directly affects the detection effect of the neural network [31]. In the text extraction model on CNN, the common method of text direction quantification is to supplement and crop the text after preprocessing and concatenate the word vector corresponding to each word in the text to obtain each word in the assembled text to obtain the direct quantification of the text [32]. For the Weibo object detection model on convolution depth, when preprocessing the Weibo text, the text less than the threshold length is filled with zero value, and the text greater than the threshold length is cropped. And then, the word vector of each word is spliced, and the obtained Weibo text information is vectorized, and the vectorized representation process of the entire Weibo text is shown in Figure 5.

The training corpus in Figure 5 is the Weibo text corpus and real-time news corpus. Text preprocessing includes operations such as word segmentation, word extraction, and removal of low-frequency words from the text information. Filling and cropping: zero-value padding for the length less than and cropping for the part whose length are greater than the text length threshold. Then, the trained word vector is used to assign the processed text to obtain the vectorized representation of the Weibo text.

#### 3.5.4. Optimized Training of the Neural Network

Dropout layer: it is the characteristic layer for overfitting in the neural network. In the process of forwarding propagation of the network, some activated neurons are randomly discarded, which can increase the necessary redundancy of the network. Meanwhile, in the case of loss of activated neurons, the model is allowed to maintain the correct classification, which reduces the problem of overadjustment so that the obtained model and training data will not be too much [33].

The formation of CNN is the principle of network training for each layer. The initial weight of the CNN training layer is random, and the backpropagation algorithm is used to adjust the corresponding weight value [34]. The reverse algorithm is divided into four parts: forward propagation, backpropagation, comparison and update of the loss function, and weight. The initial filter cannot effectively extract features. The loss function usually uses the average square error, that is, the semiaverage square error, to calculate the error between the result of the propagation phase prediction and the propagation of the true mark. Backpropagation determines important weights and adjusts the weights to reduce the overall error of the model. The detection process of the Weibo object detection algorithm on DCNN is shown in Table 1.

The article "Security Analysis of Social Network Topic Mining Using Big Data and Optimized Deep Convolutional Neural Network" was published in 2022. Journal: Comput Intell Neurosci.

#### 3.5.5. Implementation and Research of Weibo Security Topic Detection Model on DCNN

When building a new DCNN model, a large amount of data training set and related interference data set are usually needed for model training. It aims to detect and identify Weibo security topics. Therefore, the training data set and the interference data set are image data. The size of the image is defined as 224 *∗* 224 pixels. The DCNN model is designed on this basis. Information on Weibo can usually be grouped into topic templates, like the task of classifying text. The most important step is to obtain the expression characteristics of Weibo topics [35]. Traditional topic detection methods use unary language models to represent Weibo topics, often ignoring potential syntactic and semantic information. Using the DCNN model, it is possible to learn the grammatical and semantic information of Weibo more deeply, make the features of Weibo more accurate, and improve the accuracy of Weibo topic detection. The subject detection framework on DNN is shown in Figure 6.

Weibo is first preprocessed and trained through the network, and word vectors are obtained to represent each piece of Weibo information. Second, the vector matrix of Weibo keywords enters the DCNN, and the result shows that the feature vector of each Weibo can be obtained by training the DCNN. The word vector representation of Weibo is shown in the following equations:

(10) $$\begin{array}{c} P=w1\cdots ws\text{.} \end{array}$$

*P* is a Weibo sentence. The short Weibo text can be seen as a sentence. *w*1 ⋯ *ws* is the word vector of each word in Weibo.

The Weibo word vector matrix is input into the DCNN, and the feature map of the Weibo is obtained through the convolutional layer including the filter.

(11) $$\begin{array}{c} c=\left[c_{1},c_{2},\ldots \ldots c_{n-h+1}\right]. \end{array}$$

*Ci* is the feature of the Weibo topic after filtering the results.

(12) $$\begin{array}{c} ci=f\left(W\cdot X_{i.j+h-1}+b\right)\text{,} \end{array}$$

where *h* is the window size of the topic filter and *b* is the paranoid value.

This study aims to analyze and compare the performance of DCNN's Weibo security topic detection model. Irregular data detection algorithms are used in the three-dimensional data system to make judgments on topic extraction performance. Topic security is detected on the Internet. The algorithm flow of data detection and transmission based on Weibo text and semantic feature extraction is shown in Table 2.

The article "Security Analysis of Social Network Topic Mining Using Big Data and Optimized Deep Convolutional Neural Network" was published in 2022. Journal: Comput Intell Neurosci.

### 3.6. Simulation Experiment

The experiment uses Weibo as a social network instance and uses the data crawled in Weibo as a verification data set for judging the security of social network topic content. The experimental data is divided into 10 in total. There are 1,000 documents in text language, including technology, art, life, entertainment, economy, education, electronics, energy, environment, and history. The detailed distribution is shown in Table 3. Since some categories of text are relatively small and not representative, categories with more than 100 texts are selected for experimentation. Among them, the training data is 40%, and the test data is 60%.

To verify the proposed algorithm more objectively, supervised learning training is carried out in combination with the click tag of the Weibo content, and topic subtags are created for the click tag manually to further improve the accuracy of the evaluation. The algorithm uses MATLAB software to carry out data analysis and simulation experiments to verify the algorithm performance of the improved DCNN. In the experiment, the number of iterations of the neural network algorithm is 120, the simulation time is 2000 seconds, and the batch is 128. The objective function is optimized using MATLAB software. The environmental parameter settings of the software are shown in Table 4.

The constructed DCNN Weibo security topic mining and detection model is compared with neural network models proposed in other related fields, including CNN, DNN, and AlexNet, to evaluate the detection accuracy of the model. The prediction accuracy of the model is analyzed from the angles of accuracy, precision, recall, and *F*1 value. In addition, the above models are compared and analyzed, and the average transmission rate and average delay time of the models are used to evaluate the secure transmission performance of social network data.

## 4. Results and Discussion

### 4.1. Analysis of Detection Performance of Different Models

To study the detection effect of the improved DCNN on social network security topics, the detection results of the model are analyzed from the perspectives of accuracy, precision, recall, and *F*1 value. The indicators of the proposed model are compared with models, such as CNN, DNN, and AlexNet. And the results are shown in Figures 7–10. Further compare the training time and testing time required for each model, as shown in Figures 11 and 12.

The article "Security Analysis of Social Network Topic Mining Using Big Data and Optimized Deep Convolutional Neural Network" was published in 2022. Journal: Comput Intell Neurosci.

As shown in Figures 7–10, the constructed system model is compared with the neural network model proposed by scholars in other related fields from the perspectives of accuracy, precision, recall, and *F*1 value. It is found that the recognition accuracy of the constructed model can reach 96.17% after 120 iterations of the model, which is at least 5.4% higher than other models. Meanwhile, the accuracy, recall, and *F*1 value of the intrusion detection model are 88.57%, 75.22%, and 72.05%, respectively. Compared with other algorithms, the model's accuracy, recall, and *F*1 value are higher, at least 3.1% higher than other models. Therefore, compared with the network security detection model proposed by other scholars in related fields, the security detection model of the improved social network platform has better recognition and prediction accuracy.

This research further compares and analyses the training time and test time required for each algorithm, and the results are shown in Figures 11 and 12. As the number of iterations increases, the required training time and testing time show a trend of first decreasing and then basically stable; that is, convergence is achieved. In addition, the training time and testing time of the improved DCNN network security detection model stabilized at 65.86 s and 27.90 s, respectively. Compared with the models proposed by other scholars, the prediction time of the improved DCNN network security detection model is significantly shortened. This may be because the improved DCNN network security detection model can enhance the generalization ability and accelerate the convergence speed of the model training process. Therefore, for the mining and analysis of social network security topics, the improved DCNN network security detection model can obtain higher prediction results in a shorter time.

### 4.2. Data Transmission Security Performance Analysis of Different Network Models

From the aspects of the average transmission rate and data transmission delay of network data security transmission performance, the improved DCNN network security topic detection model is further compared with AlexNet, CNN, and DNN. The results are shown in Figures 13 and 14.

By comparing the network data security transmission performance of each model under different transmission data, with the increase of transmission data, the average delivery rate of network data shows an upward trend.  Figure 13 shows that the data message transmission rate of the improved DCNN network security detection model is not less than 80%. In terms of average delay, the average delay decreases with the increase of transmitted data. The average delay of the improved DCNN network security detection model is stable at about 360 ms, as shown in Figure 14. Therefore, from the perspective of different data transmission, the improved DCNN security detection model has the characteristics of lower delay and shows good network data security transmission.

The article "Security Analysis of Social Network Topic Mining Using Big Data and Optimized Deep Convolutional Neural Network" was published in 2022. Journal: Comput Intell Neurosci.

### 4.3. Discussion of Results

The test results of the model are analyzed from the perspectives of accuracy, recall, and *F*1 value. The accuracy, recall, and *F*1 values of the intrusion detection model are 88.57%, 75.22%, and 72.05%, respectively. Compared with other algorithms, this model has higher accuracy, recall, and *F*1 value. It is at least 3.1% higher than other models. The data message transmission rate of the improved DCNN network security detection model is not less than 80% compared with AlexNet, CNN, and DNN. The average delay decreases as the transmitted data increases. Li et al. [36] conducted gesture recognition research based on CNN, optimized the classification function of CNN, and improved the effectiveness and robustness of the entire model. Geirhos et al. [37] researched shortcut learning in DNNs. The study shows that fast learning is an important common feature of deep learning systems. Jiang et al. [38] researched the design of DNNs for photonic devices and discussed the network training process, the division of different network types and architectures, and the process of dimensionality reduction. The research has practical reference value for the simulation and design of the photonic system [39–45]. In summary, the results of CNN and DNNs have been applied in various fields in the research work of predecessors [46–49]. The difference between this study and previous studies is the use of DCNN to complete the analysis and search of social network security issues [50–52]. Meanwhile, the LSTM algorithm in the memory wisdom algorithm is used for the extraction of Weibo topic information. This is of great significance to the improvement of the security transmission performance of social network data.

## 5. Conclusion

With the rapid development of information technology, information security issues in social networks have become increasingly severe, and it is urgent to detect network attacks or intrusions. This study extracts the vector data of Weibo-related security topics through the research of social network security issues, combined with the mining and data analysis of network security topics. Weibo security topics are detected based on Latent Dirichlet Allocation and DNN. Meanwhile, DCNN's Weibo security topic detection model is implemented and used to improve the CNN. Combined with the DNN, the improved DCNN security detection model is implemented to ensure the safe operation of social networks. Finally, through the performance analysis of simulation experiments, the improved DCNN network security detection model predicts accuracy and precision rates of 96.17% and 88.57%, respectively, showing high prediction performance and good data transmission performance. The experimental results can be as follows: the security of social networks provides experimental evidence. However, some shortcomings still exist. Firstly, the dynamic growth of Weibo in real life is very fast, and the establishment of a fast, iterative text data representation is an important factor to be considered in the subsequent research. Secondly, there are not only texts on Weibo, but also a large amount of multimedia information, such as images and videos. How to mine the security topics of this part of the information is a difficult point in search research. Therefore, it is necessary to consider more factors in this aspect in future research.

The article "Security Analysis of Social Network Topic Mining Using Big Data and Optimized Deep Convolutional Neural Network" was published in 2022. Journal: Comput Intell Neurosci.

## Figures and Tables

**Figure 1:** Mining topic data on social networks.

**Figure 2:** Weibo topic feature extraction structure diagram.

**Figure 3:** Framework diagram of Weibo security topic mining and detection.

**Figure 4:** Neural network structure for obtaining topic depth semantics.

**Figure 5:** The vectorized representation process of Weibo text.

**Figure 6:** CNN text classification diagram.

**Figure 7:** Comparison of the accuracy of different models.

**Figure 8:** Comparison of precision of different models.

**Figure 9:** Comparison of recalls of different models with an increasing number of iterations.

**Figure 10:** Comparison of *F*1 values of different models with an increasing number of iterations.

**Figure 11:** Comparison of training time of different models.

**Figure 12:** Comparison of test time of different models.

**Figure 13:** Comparison of the average data transmission rate of each model network under different transmission volumes.

**Figure 14:** Comparison of average network data delay of each algorithm under different transmission volumes.

**Table 1:** Weibo topic detection on DNN.

Weibo topic detection steps on DCNN

Input: Weibo text data of the topic to be detected
(1) Text preprocessing of Weibo topic data
(2) Build a DCNN model and initialize the network
(3) Use the word vector representation of the Weibo used for training as the input of the DCNN to train the DCNN model
(4) For the Weibo to be detected, use the trained DCNN model to predict, obtain the topic label, and complete the Weibo topic detection
Output: Weibo hashtag

**Table 2:** Data security detection algorithm flow based on semantic feature extraction.

(1) Algorithm: DCNN
(2) **Input:** the raw points of *P*={*p*_1_, *p*_2_,…, *p*_*n*_}
(3) **Output:** the ground surface points *p*_*g*_
(4) **Parameters:**b_0_, b_*k*_, H, *μ*, *λ*, *C*_*th*_, *V*_*s*_*n*__
(5) Mapping all the point cloud data into the polar grid Gri d (*m*, *k*)=PolarGri dM ap(P, b_0_, b_*k*_, H, *μ*, *λ*)
(6) Initialization *p*_*g*_=∅
(7) **For***s*=0 : *m* − 1 do
(8) **For***j*=0 : *k* − 1 do
(9) Gri d (S_*x*_, b_1_)={p_*i*_=(*x*_*i*_, *y*_*i*_, *z*_*i*_)}
(10) The *z*-coordinate value of the point plus the laser installation Gri d (S_*x*_, b_1_)={p_*i*_=(*x*_*i*_, *y*_*i*_, *z*_*i*_+*H*)}
(11) Order the points in the grid Gri d (S_*x*_, b_1_) at height
(12) *n* = 1
(13) **IF**p_1_^2^ > *C*_*w*_
(14) return
(15) **Else**
(16) **While**Δ*z*=p_*j*+1_ − p_*i*_^2^ < *V*_*t*a_
(17) *N* = *n *+* *1;
(18) **End while**
(19) **End IF**
(20) **End For**
(21) **End For**
(22) **Return***p*_*g*_

**Table 3:** The text used in the experiment.

Number	Category	Quantity	Proportion (%)
1	Technology	75.5	7.55
2	Art	47.5	4.75
3	Life	65.3	6.53
4	Entertainment	138.4	13.84
5	Economy	124.1	12.41
6	Education	104.1	10.41
7	Electronics	163.2	16.32
8	Energy	104.4	10.44
9	Environment	107.6	10.76
10	History	20.2	2.02

The article "Security Analysis of Social Network Topic Mining Using Big Data and Optimized Deep Convolutional Neural Network" was published in 2022. Journal: Comput Intell Neurosci.

**Table 4:** Parameter settings of simulation experiment environment.

	Test environment parameters
System structure	B/S
CPU	Intel Core i5-6300HQ
Main frequency	2.3 GHz
RAM	8.00 GB
Development language	Java
Server database	Tomcat MySQL

## Data Availability

The raw data supporting the conclusions of this article will be made available by the authors, without undue reservation.
